This article has been retracted.

# Clinical Efficacy of Osimertinib in Patients with Advanced Non-Small Cell Lung Cancer and Its Effect on Serum CEA and VEGF Expression

**DOI:** 10.1155/2022/3032087

**Published:** 2022-05-25

**Authors:** Huanyuan Wang, Xiangwu Zhou, Zhaozhen Wang, Tianzhu Lu, Baoliang Li, Sicong Jiang

**Affiliations:** ^1^Department of Thoracic Surgery, Jiangxi Cancer Hospital of Nanchang University, Nanchang 330029, China; ^2^Department of Thoracic Surgery, Medical College of Nanchang University, Nanchang 330006, China; ^3^Department of Clinical Medicine, Jiangxi Health Vocational College of China, Nanchang, Jiangxi, China; ^4^Department of Radiation Oncology, Jiangxi Cancer Hospital of Nanchang University, Nanchang 330029, China; ^5^Guangdong Provincial Key Laboratory of Orthopedics and Traumatology, Orthopaedic Research Institute/Department of Spinal Surgery, The First Affiliated Hospital of Sun Yat-Sen University, Guangzhou 510080, China; ^6^Division of Thoracic and Endocrine Surgery, University Hospitals and University of Geneva, Geneva 1211, Geneva 4, Switzerland

## Abstract

**Objective:**

To assess the clinical efficacy of osimertinib in patients with advanced non-small cell lung cancer and its effect on serum carcinoembryonic antigen (CEA) and vascular endothelial growth factor (VEGF) expression.

**Methods:**

Between July 2018 and January 2020, 80 patients with advanced non-small cell lung cancer were assessed for eligibility and recruited. The patients were assigned at a ratio of 1 : 1 to receive either the PC regimen (pemetrexed + cisplatin) (conventional group) or osimertinib (experimental group). The primary endpoint was the clinical efficacy, and the secondary endpoints were the adverse events, expression of serum CEA and VEGF, and 2-year survival.

**Results:**

Osimertinib was associated with a significantly higher response rate and disease control rate versus pemetrexed plus cisplatin (*P* < 0.05). Osimertinib resulted in a significantly lower incidence of adverse events versus the PC regimen (*P* < 0.05). Patients given osimertinib had significantly lower levels of CEA and VEGF versus those given pemetrexed plus cisplatin (*P* < 0.05). Osimertinib was associated with a significantly higher 1-year and 2-year survival rate versus pemetrexed plus cisplatin

**Conclusion:**

Osimertinib could inhibit the expression of serum CEA and VEGF in patients with advanced non-small cell lung cancer and reduce the adverse events with significant efficacy, so it is worthy of clinical promotion and application.

## 1. Introduction

Lung cancer is currently the most prevalent malignancy with the highest mortality rate worldwide, among which non-small cell lung cancer (NSCLC) accounts for approximately 78% [1]. Due to the absence of specific signs and symptoms in the early stages of NSCLC, about 70% of cases have progressed to an advanced stage at the time of diagnosis, where patients showed an excessively poor 5-year survival [2]. The Japanese Cancer Institute recommends chemotherapy treatment for patients with advanced NSCLC without surgical indication, of which PC regimen (pemetrexed + cisplatin) is well-recognized [3] and can efficiently promote apoptosis of tumor cells. However, numerous clinical studies have shown that the PC regimen (pemetrexed + cisplatin) is associated with considerable adverse events and suppression of immune function [4], which is detrimental to the functional recovery of patients [5]. It has been confirmed that epidermal growth factor receptor gene mutations are present in 35%–45% of NSCLC patients in China, and the 1st and 2nd generation EGFR complex kinase inhibitors are available for targeted treatment of NSCLC, which substantially prolongs the survival of patients [6]. Nevertheless, its acquired resistance results in disease progression after 6–12 months of treatment, and about 58% of all drug resistance is attributed to T790M mutations [7]. Osimertinib belongs to the 3rd generation EGFR-TKIs and is the only drug currently available for the treatment of NSCLC with EGFR-T790M mutation-positive and resistance to 1st generation EGFR-TKIs [8]. Relevant animal experiments have revealed that osimertinib could inhibit tumor growth, improve immunity, and prolong the survival of NSCLC mice [9]. There are few relevant trials on the application of osimertinib in clinical practice in China. Accordingly, 80 patients with advanced non-small cell lung cancer were recruited to assess the clinical efficacy of osimertinib in patients with advanced non-small cell lung cancer and its effect on serum CEA and VEGF expression to provide a reference basis for clinical practice. The novelty of this study is the use of osimertinib, which is a 3rd generation EGFR-TKIs, and is the only current treatment for EGFR-T790M mutation-positive NSCLC that is resistant to 1st generation EGFR-TKIs.

## 2. Materials and Methods

### 2.1. Baseline Data

Between July 2018 and January 2020, 80 patients with advanced non-small cell lung cancer were assessed for eligibility and recruited. The patients were assigned to either a conventional group (*n* = 40) or an experimental group (*n* = 40). Patients in the conventional group were aged 53–82 years, and those in the experimental group were aged 54–82 years. The studies involving human participants were reviewed and approved by our hospital, no. JX3971. The patients provided their written informed consent to participate in this study.

### 2.2. Inclusion and Exclusion Criteria

Inclusion criteria are as follows: (1) all patients were diagnosed by MRI imaging and pathology, met the diagnostic criteria for non-small cell lung cancer as per the Clinical Practice Guidelines for Non-Small Cell Lung Cancer, were diagnosed as stage IIIA, IIIb, and IV as per the international lung cancer staging criteria, with T790M mutation by genetic testing, or received osimertinib after disease progression of first-line/multiline therapy (after application of the first generation of EGFR-TKIs); (2) with an expected survival of >3 months and a Karnofsky performance status (KPS) score of >60 points; (3) without symptoms of systemic failure.

Exclusion criteria are as follows: (1) patients with severe liver and kidney injury, cardiovascular diseases, and autoimmune diseases; (2) with extensive systemic metastases and cachexia; (3) with poor compliance, intolerance of treatment or withdrawal of consent; (4) with severe psychiatric diseases; (5) with other targeted drugs against T790M mutation before the use of osimertinib.

### 2.3. Methods

The conventional group was given the conventional PC regimen chemotherapy: pemetrexed (Nanjing Pharmaceutical Factory Co. Ltd., National Drug Administration H20080177, specification 0.5 g) 500 mg/m^2^ was given intravenously on day 1. Cisplatin (Guangdong Lingnan Pharmaceutical Co. Ltd., State Drug quantification H20183341, specification 10 mL:10 mg) 20 mg/m^2^ was given 30 min after the pemetrexed administration, days 1–5. The experimental group was given oral osimertinib (Sweden-AstraZeneca AB, State Drug Administration J20180027, specification 80 mg), at a dose of 80 mg/d. One course of treatment was 21 d. Both groups of patients were treated for 4 courses.

### 2.4. Endpoints

(1) Efficacy assessment criteria: at the 4th week after treatment, short-term efficacy was evaluated with reference to the efficacy assessment criteria of solid tumors. Complete response (CR): patients' lesions disappeared and lasted for at least 4 weeks; partial response (PR): the patient's tumor volume was reduced by > 50% and lasted for at least 4 weeks; stable disease (SD): the patient's tumor volume increased by 25% or reduced by < 50%; progressive disease (PD): the patient's tumor volume increased by > 25%. Treatment response rate (RR) = CR + PR; disease control rate (DCR) = CR + PR + SD. (2) Adverse events: adverse events included white blood cell decline, liver function damage, rash, pruritus, and neutropenia, and the incidence of adverse events of calculated. (3) Serum indices: before and after treatment, 5 mL of fasting venous blood was collected from two groups of patients, centrifuged at 3000 r/min for 10 min, and the serum was collected to determine the levels of carcinoembryonic antigen (CEA) and vascular endothelial growth factor (VEGF) by the enzyme-linked immunoassay, with the kits provided by Beijing Wantai Biological Pharmaceutical Co. The normal reference value of CEA was ≤5.90 *μ*g/L, and the normal reference value of VEGF was <127 pg/mL.

### 2.5. Statistical Analysis

SPSS 21.0 was used for data analyses. The measurement data were expressed as ($\bar{x}$ ± s) and processed using the independent samples *t*-test. The count data were expressed as the number of cases (rate) and processed using the chi-square test. Survival analysis was performed using Kaplan–Meier analysis. Differences were considered statistically significant at *P* < 0.05.

## 3. Results

### 3.1. Baseline Data

The two groups showed similar baseline data (*P* > 0.05). (Table 1).

### 3.2. Clinical Efficacy

Osimertinib was associated with a significantly higher response rate and disease control rate versus pemetrexed plus cisplatin (*P* < 0.05) (Table 2).

### 3.3. Adverse Events

Osimertinib resulted in a significantly lower incidence of adverse events versus the PC regimen (*P* < 0.05) (Table 3).

### 3.4. Serum CEA and VEGF

Patients given osimertinib had significantly lower levels of CEA and VEGF versus those given pemetrexed plus cisplatin (*P* < 0.05) (Table 4).

### 3.5. 2-Year Survival

The two groups had similar 6-month survival (94.29% vs. 91.43%) (*X*2 = 0.235, *P* = 0.671). Patients receiving osimertinib showed a higher 1-year and 2-year survival (77.14% and 54.29%) versus those given pemetrexed plus cisplatin (60.00% and 34.29%) (*X*2 = 4.058, *P*=0.044, *X*2 = 4.644, *P*=0.031).

## 4. Discussion

In recent years, the incidence of non-small cell lung cancer has shown an increasing trend [10], and clinical data show that about 50% of cases with NSCLC are over 60 years old, and nearly 30% of patients are over 70 years old [11]. Elderly patients are mostly accompanied by underlying diseases, and the lack of typical symptomatic manifestations in the early stage of NSCLC usually results in an advanced stage of disease by the time patients develop symptoms such as irritating dry cough, chest tightness, chest pain, and hoarseness [12]. Clinically, surgery is considered little effective for advanced NSCLC, so chemotherapy and radiotherapy are the current mainstays of treatment [13]. PC regimen (pemetrexed + cisplatin) is the treatment of choice for advanced lung cancer, as it can effectively suppress tumor development. However, clinical studies have revealed the association of the PC regimen with impaired immune function, significant adverse events, and poor prognosis [14]. Thus, there exists a need to explore more efficient treatment protocols [15]. Molecular targeted therapy mainly refers to the use of targeted drugs to act on key molecules in the signaling pathways to inhibit the proliferation and invasion of malignant tumors with high safety [16]. Osimertinib is the latest generation targeted drug that acts on the EGFR signaling pathway and competitively binds to EGFR to inhibit complex kinase activation, thereby blocking the EGFR signaling pathway, which consequently inhibits tumor cell proliferation and metastasis and promotes tumor cell apoptosis [17]. It is clinically available in patients with Troche.

A related study by Schmid et al. evaluated the efficacy of osimertinib in advanced non-small cell lung cancer, in which the disease control rate was 85% in 27 patients with confirmed positive EGFR T790 M mutations, and further analysis of the efficacy of osimertinib in patients with T790M-positive brain metastases revealed no significant difference in the comparison with those without brain metastases, indicating that osimertinib is equally effective in patients with advanced non-small cell lung cancer with brain metastases [18]. In the present study, osimertinib was associated with a significantly higher response rate and disease control rate versus pemetrexed plus cisplatin, which is consistent with the previous research results, suggesting a promising clinical efficacy of osimertinib for patients with non-small cell lung cancer. Moreover, osimertinib resulted in a significantly lower incidence of adverse events versus the PC regimen, indicating a higher safety profile of osimertinib [19]. Clinical studies have shown that patients with non-small cell lung cancer have higher than normal levels of CEA, the expression of which can visually reflect tumor cell activity, and that VEGF, a heparin-binding growth factor specific for vascular endothelial cells, can induce neovascularization in patients. The results of Wu et al. showed that tumor tissue growth requires neovascularization to provide oxygen and nutrients for maintenance [20]. Herein, the patients given osimertinib had significantly lower levels of CEA and VEGF versus those given pemetrexed plus cisplatin, indicating that osimertinib can effectively downregulate serum CEA and VEGF levels in patients with non-small cell lung cancer, which thus mirrors its inhibition of tumor cell growth or metastasis. The reason for this may be attributed to the inhibition of EGFR-T790M mutation-positive or cancer cell spread by osimertinib [21]. VEGF is a vascular endothelial cell-specific heparin-binding growth factor that induces vascular neovascularization in vivo. Studies have shown that tumor tissue growth must be maintained by neovascularization to provide oxygen and nutrients. Therefore, monitoring VEGF expression can visually reflect the development of tumor tissue. Osimertinib has been shown to be effective in the short- and long-term treatment of NSCLC, with suppression of CEA and VEGF expression, prolonged survival, and tolerable side effects. However, it is worth noting that this regimen still exhibits a certain incidence of failure in the treatment of advanced NSCLC due to resistance mechanisms such as C797S mutation, activation of multiple bypass pathways, and epithelial-mesenchymal transition, so a more effective treatment regimen remains to be explored. The limitation of this study is the absence of drug resistance research, and more relevant data will be obtained in the future during long-term follow-up to obtain more detailed data. Compound Kushen injection is extracted and refined from bitter ginseng and white tulip, rich in alkaloids such as bitter ginseng alkaloids and oxidized bitter ginseng alkaloids, which are widely used in antitumor, anti-hepatitis B virus, anti-inflammatory, and antiallergy applications. As bitter ginseng alkaloids can inhibit the proliferation of lung cancer cells and induce their apoptosis, Kushen injection can be introduced to the treatment of NSCLC to explore more effective treatment regimens.

## 5. Conclusion

Osimertinib could inhibit the expression of serum CEA and VEGF in patients with advanced non-small cell lung cancer and reduce the adverse events with significant efficacy, so it is worthy of clinical promotion and application.

## Figures and Tables

**Table 1:** Comparison of baseline data (*n* (%)).

	Conventional group (*n* = 40)	Experimental group (*n* = 40)	*t* or *x*^2^	*P* value
*Gender*				
Male	24	26	0.213	0.644
Female	16	14		

Mean age (year)	66.87 ± 5.34	66.93 ± 5.36	−0.05	0.96
*Smoking*				
Yes	27	28	0.058	0.809
No	13	12		

*TNM staging*				
IIIA	18	20	0.075	0.785
IIIB	13	12		
IV	9	8		

*Pathological type*				
Adenocarcinoma	37	38	0.213	0.644
Adenosquamous carcinoma	3	2		

**Table 2:** Comparison of clinical efficacy (*n* (%)).

	Conventional group (*n* = 40)	Experimental group (*n* = 40)	*x* ^2^	*P* value
CR	8	13		
PR	11	20		
SD	7	3		
PD	14	4		
RR	19 (48%)	33 (83%)	10.769	0.001
DCR	26 (65%)	36 (90%)	7.168	0.007

**Table 3:** Comparison of adverse events (*n* (%)).

	Conventional group (*n* = 40)	Experimental group (*n* = 40)	*x* ^2^	*P* value
White blood cell decline	5	0		
Liver function impairment	4	0		
Skin rash	2	4		
Pruritus	1	3		
Neutropenia	3	0		
Total incidence (%)	15 (38%)	7 (18%)	4.013	0.045

**Table 4:** Comparison of serum CEA and VEGF levels ($\bar{x}$ ± *s*).

Groups	*n*	CEA (U/mL)		VEGF (pg/mL)	
		Before treatment	After treatment	Before treatment	After treatment
Conventional group	40	10.41 ± 1.34	8.26 ± 0.59	242.37 ± 20.26	168.39 ± 15.51
Experimental group	40	10.28 ± 1.37	5.17 ± 0.61	242.35 ± 20.30	121.42 ± 13.41
*t*	—	0.429	23.028	0.004	14.489
*P* value	—	0.669	<0.001	0.997	<0.001

## Data Availability

The datasets used during the present study are available from the corresponding author upon reasonable request.
